The article "Effect of soft tissue thickness on accuracy of conventional and digital implant impression techniques" was published in 2024. Journal: BMC Oral Health.

# Effect of soft tissue thickness on accuracy of conventional and digital implant impression techniques

**DOI:** 10.1186/s12903-024-05037-4

**Published:** 2024-10-30

**Authors:** Eman Mostafa Awad, Mohamed Maamoun ElSheikh, Azza Abd el moneim El-Segai

**Affiliations:** 1 Ministry of Health and Population, Cairo, Egypt; 2 Faculty of Dentistry, Tanta University, Tanta, Egypt

**Keywords:** Implant depth, Conventional impression, Digital impression, Accuracy of impression

## Abstract

**Background:**

Placing implants deep sub-gingivally may affect the accuracy of implant impression techniques and the fit of final restoration.

**Purpose:**

The aim of this in-vitro study was to evaluate the effect of soft tissue thickness on accuracy of conventional and digital implant impression techniques.

**Methods:**

Four parallel implant analogues (A, B, C, D) placed in each of two epoxy resin models representing edentulous mandible covered by flexible polyurethane material with two different thickness two mm and four mm. A total of sixty impressions performed, thirty impressions for each model divided into four groups (*n* = 15 per group) GI (C2mm) open tray impression with two mm implant depth, GII (C4mm) open tray impression with four mm implant depth, GIII (D2mm) digital impression with two mm implant depth, GIV (D 4 mm) digital impression with four mm implant depth. Impressions from open tray technique were poured to get stone casts while impressions from digital scanning technique were printed as three-dimensional printed casts. The six inter-implant distances between analogues were measured using Co-ordinate measuring machine, deviations compared to reference models were calculated. Data was collected, tabulated and statistically analyzed using One-way ANOVA test to detect significances between groups.

**Results:**

For conventional impressions there was significant difference between C2mm/C4mm (*P* < 0.001) regarding interimplant distance, while in digital impressions there was no significant difference between D2mm/D4mm AB(*p* = 0.110), BC(*p* = 0.066), CD(*p* = 0.710), AD(*p* = 0.084), AC(*p* = 0.067) and BD(*p* = 0.072). There was significant difference between conventional and digital impression techniques C2mm/D2mm, C4mm/D4mm (*P* < 0.001).

**Conclusion:**

Within the limitations of this in-vitro study digital impressions provide more accurate outcomes with implants placed deeper subgingivally than conventional impressions.

**Trial registration:**

Retrospectively registered.

## Background

For long-term implant-supported prostheses success, one of the most crucial factors is passive fit [1]. Absolute passive fit of superstructure and implant is scarcely possible as errors seems to be unavoidable because of numerous steps in processing and manufacturing in implant restoration [2, 3]. Non passive fit may lead to many complications mechanical and biological [4, 5]. When considering passive fit, accuracy of the impression procedures becomes a serious problem [6–8].

The article "Effect of soft tissue thickness on accuracy of conventional and digital implant impression techniques" was published in 2024. Journal: BMC Oral Health.

There are two main implant impression techniques that are used to transfer the intra-oral spatial relation of the implants to the working cast. The first is the conventional impression technique, which has two types: closed tray technique and open tray technique (splinted or unsplinted). The second is the digital impression technique, which has two types: direct intraoral scan and indirect extraoral scan [9].

In conventional impressions techniques, splinting or unsplinting, type of impression tray^,^ impression materials, soft tissue thickness and depth of the implant, implant or abutment level impression, impression copings modifications, implant angulations and numbers, connection of implants, machining tolerance and the interval between making the impression and pouring are factors that affect implant impressions techniques accuracy [10–12].

While in digital impressions inter implant distances, scan body type, implant angulation, depth of the implant, connection of implant, experience of operator, types of oral scanners, the congruence between mesh of scanbodies (SBs) and implant library files (LF), scanning strategies and types of digital coping are factors that affect accuracy implant impressions [13–15].

However, in some clinical situations, the availability of bone, aesthetic concerns, and/or the thickness of the soft tissue necessitate placing the implant more subgingivally. Consequently, a greater portion of the scanbody or impression coping is positioned beneath the gingival margin. Consequently, the supra-gingivally exposed area of the coping or scan body reduces [7]. The accuracy of the impression is impacted by this decrease in the scan body and impression coping surface. Few research, according to the authors, have examined the impact of subgingival implant placement on the dimensional accuracy of impressions and the castings that are produced [7, 11, 16].

Because of the above-mentioned shortcomings this in-vitro study aimed to evaluate the effect of soft tissue thickness (subgingival depth of implant) on accuracy of conventional versus digital impression technique for implant restorations.

Two null hypotheses were tested the first one was tested is there were no significant differences in accuracy of implant level impressions of different tissue thickness and subgingval depths of implant placement. And the second was no significant difference between conventional impressions technique and digital impressions technique.

The article "Effect of soft tissue thickness on accuracy of conventional and digital implant impression techniques" was published in 2024. Journal: BMC Oral Health.

## Methods

As definitive models (reference models), two fully edentulous mandibular epoxy resin models (Ramses Medical Products Factory, Alex, Egypt) were covered in two distinct flexible polyurethane material thicknesses. There were four implant analogues for Model (1) with a flexible polyurethane layer thickness of 2 mm and Model (2) with a layer thickness of 4 mm (Nucleoss, Menderes/Izmir, Turkey). Two implant analogues were positioned perpendicular to the base of the model, parallel to each other, at the anterior canine regions and posterior first molar regions, respectively.

As shown in Fig. 1, the four implants on each model were assigned a letter. The two models were prepared for the impression procedures and had labels applied. In order to create two stone casts and thirty identical custom trays for each cast, the two reference models were duplicated and custom trays were then fabricated. For the two reference models (*n* = 15 per group), two distinct impression procedure techniques were applied with four distinct groups as follows: A-Conventional impression method (direct unsplinted). B. The digital impression method (Table 1). The impressions for groups C2 and C4 were made using conventional methods. Four open tray impression copings from (Nucleoss, Menderes, Izmir, Turkey), which were appropriate for implant analogues, were first roughened on the outside with 50 μm aluminum oxide powder, subsequently, utilizing a specialized torque wrench calibrated at 10 Ncm, the copings were tightened to the implant equivalents. Brushed, after which a thin layer of adhesive was applied to the imprint copings and fitting surface of the custom tray. The adhesive was then allowed to dry for 15 min before the impression was made. Figure 2 The additional silicone impression material (Elite^®^ Stone, Zhermack GmbH Deutschland.) was auto-mixed, injected to cover the impression copings, inserted into the tray and seating of the tray in its position with finger pressure then applying 1.5 kg metal block to standardize pressure during setting of the material.

**Fig. 1:** Six distances between four implant analogues

**Fig. 2:** **(A)** Sandblasted impression coping. Figure 1.**(B)** Short part of impression coping inserted in flexible polyurethane material. Figure 1.**(C)** Increased part of impression coping inserted in 4 mm flexible polyurethane material

**Table 1:** Description of the studying groups

Impression technique	thickness of flexible polyurethane layer	Groups	Number of samples
Conventional Impression	2 mm	Group I (C2mm)	15
Conventional Impression	4 mm	Group II (C4mm)	15
Digital Impression	2 mm	Group III (D2mm)	15
Digital Impression	4 mm	Group IV (D4mm)	15

Excess was taken out of the impression coping screws after setting. After unscrewing and extracting the screws, the tray was taken out of the model. After connecting the implant analog to the hex on the bottom and tightening the screw pins, the screws were reinserted into the impression copings from the top. The impression was examined for accuracy, and if necessary, a new one was created. Digital impressions for groups (D2mm) and (D4mm) were taken, in accordance with the manufacturer’s instructions, PEEK impression scanbodies (Nucleoss, Menderes/Izmir, Turkey) that matched the analogues of T6 implants were screwed and tightened. To obtain accurate data, spray the scanbodies with scan powder (Dentify GmbH, Scheffelstr. 22, 78234 Engen, Germany) in accordance with the manufacturer’s instructions before scanning Fig. 3.

The article "Effect of soft tissue thickness on accuracy of conventional and digital implant impression techniques" was published in 2024. Journal: BMC Oral Health.

**Fig. 3:** Scanbody connected to implant analogues of reference models

The model with the attached scanbodies was placed directly on the table of the laboratory extra oral scanner (DOF FREEDOM HD, Seoul 0479 Korea) and scanned to generate virtual reference images. Figure 4 There were no voids in the model’s scanned lingual, buccal, and occlusal surfaces and accurate imprint of implant areas indicated for accepted scanning. If the scanning did not meet these criteria was rescanned.

Two types of cast production according to technique of impression were the result, each impression taken by conventional technique were poured to obtain the corresponding model and healing abutments (Nucleoss, Menderes/ Izmir, Turkey^)^ were tightened to the implant analogues for each cast before measuring procedures on Co-ordinating measuring machine (CMM) (LK Metrology LTD, DE74 Derby, UK).

While impressions taken by digital technique were printed to get three dimensional (3D) printed casts. Healing abutments were tightened to the implant digital analogues (Nucleoss, Menderes/ Izmir, Turkey^)^ for each printed cast. and all casts were labelled before measuring on CMM.

### Measurement procedure

#### A co-ordinating measuring machine (CMM)

All reference models, stone casts from conventional technique and printed casts from digital techniques with their healing abutments were measured by (CMM). Figure 5. It was used to record three dimensional coordinates (X, Y and Z) of the implant platform centered on the reference model and their analogues on the casts that resulted. The healing abutments center consider as center point of implant position, it was located by touching eight points around the outer diameter of the abutments using a CMM probe. After locating the center of the outer diameter, the flat surface was identified as XY.The vertical distances between four healing abutments in the Z-axis were determined by measuring four locations on the upper surface of each healing abutment. These points formed a plane.

The article "Effect of soft tissue thickness on accuracy of conventional and digital implant impression techniques" was published in 2024. Journal: BMC Oral Health.

**Fig. 4:** Virtual reference images from scanning of reference models

1. The following formula was used to compute the distances (in micrometers) between the implant centers and the reference point.

2. The distance from the reference point (r) =√ X2 + Y2 + Z2.

3. By comparing the distance between the analogues in the duplicated cast with the distance in the reference model, the absolute error (Δr) was determined.

4. All measurements of stone and printed casts were collected in a table to be compare with the reference models measurements.

### Statistical analysis

IBM SPSS software package version 20.0 was used to gather, tabulate, and statistically evaluate data from measuring procedures. (IBM Corp, Armonk, NY).To confirm the distribution’s normality, the Shapiro-Wilk test was performed. The terms range, mean, standard deviation, median, and interquartile range were used to characterize quantitative data. The tests that were employed were the Post Hoc test (Tukey) for pairwise comparisons and the One-way ANOVA test for normally distributed quantitative variables when comparing more than two groups.

**Fig. 5:** Reference models, stone cast and printed cast measurement on CMM

## Result

Table 2 shown the mean values, standard deviations in micrometers for each distance, p-value, and mean difference for the six distances (AB, BC, CD, AD, AC, and BD) for each of the four study groups. There was a significant difference (p value < 0.001) in the comparison between group I (C2mm) and its reference model (1) and group II (C4mm) and its reference model (2) in six distances between implant analogues. While there was no significant difference between group IV (D4mm) and its reference model (2) and group III (D2mm) and its reference model (1) in the six distances between implant analogues, the p value was greater than 0.001.

**Table 2:** Mean & Standard deviation, p value and mean difference of 6 distances (AB, BC, CD, AD, AC, BD) of groups I (C2mm), II (C4mm), III (D2mm), IV (D4mm)

Distance	Groups	Mean ± SD.	*p*	Mean Diff.
ab	Group I	20373.9 ± 2.99	< 0.001^*^	28.93
	Group II	20253.5 ± 1.06	< 0.001^*^	49.47
	Group III	20344.1 ± 2.12	0.110	-0.93
	Group IV	20204.3 ± 2.29	0.582	0.33
bc	Group I	20757.9 ± 3.01	< 0.001^*^	-8.07
	Group II	21544.5 ± 1.36	< 0.001^*^	39.47
	Group III	20764.5 ± 2.97	0.066^*^	-1.53
	Group IV	21504.5 ± 1.06	0.110	-0.47
cd	Group I	21755.5 ± 2.45	< 0.001^*^	19.53
	Group II	20668.0 ± 1.46	< 0.001^*^	30.0
	Group III	21736.2 ± 2.04	0.710	0.20
	Group IV	20639.7 ± 2.28	0.011^*^	1.73
ad	Group I	43474.1 ± 2.71	< 0.001^*^	21.07
	Group II	43436.5 ± 1.88	< 0.001^*^	60.53
	Group III	43454.1 ± 2.36	0.084	1.133
	Group IV	43376.9 ± 2.37	0.150	0.93
ac	Group I	36054.3 ± 2.74	< 0.001^*^	25.27
	Group II	36563.3 ± 0.72	< 0.001^*^	30.33
	Group III	36030.5 ± 2.17	0.020^*^	1.47
	Group IV	36533.3 ± 1.18	0.290	0.33
bd	Group I	36934.7 ± 2.66	< 0.001^*^	22.73
	Group II	36975.9 ± 1.19	< 0.001^*^	30.87
	Group III	36913.9 ± 2.34	0.006^*^	1.93
	Group IV	36946.0 ± 1.60	0.030^*^	1.0

Data was expressed using Mean ± SD. SD: Standard deviation

p: p value for One Sample t-test comparing between Reference and each group

*: Statistically significant at *p* ≤ 0.05

The article "Effect of soft tissue thickness on accuracy of conventional and digital implant impression techniques" was published in 2024. Journal: BMC Oral Health.

### Comparing between study groups

Table 3 shown a comparison of the standard deviations (± SD), p value, and mean difference of distances in micrometers for the four groups: I (C2mm), II (C4mm), III (D2mm), and IV (D4mm) after subtracting from reference models (1, 2).

**Table 3:** Comparison between mean difference of distances in micrometer after subtraction from reference models (1, 2), standard deviations (± SD) and p value of the four groups I (C2mm), II (C4mm), III (D2mm), IV (D4mm)

	Group I (*n* = 15)	Group II (*n* = 15)	Group III (*n* = 15)	Group IV (*n* = 15)	F	*p*
AB						
Min. – Max.	25.0–34.0	47.0–51.0	-4.0–3.0	-4.0–4.0	1791.48	< 0.001^*^
Mean ± SD.	28.93 ± 2.99	49.47 ± 1.06	-0.93 ± 2.12	0.33 ± 2.29		
Sig. bet. grps.	p_1_ < 0.001^*^, p_2_ < 0.001^*^, p_3_ < 0.001^*^, p_4_ < 0.001^*^, p_5_ < 0.001^*^, p_6_ = 0.410					
BC						
Min. – Max.	-13.0 – -4.0	37.0–42.0	-6.0–3.0	-2.0–1.0	1350.64	< 0.001^*^
Mean ± SD.	-8.07 ± 3.01	39.47 ± 1.36	-1.53 ± 2.97	-0.47 ± 1.06		
Sig. bet. grps.	p_1_ < 0.001^*^, p_2_ < 0.001^*^, p_3_ < 0.001^*^, p_4_ < 0.001^*^, p_5_ < 0.001^*^, p_6_ = 0.580					
CD						
Min. – Max.	15.0–24.0	28.0–33.0	-4.0–3.0	-2.0–5.0	716.753^*^	< 0.001^*^
Mean ± SD.	19.53 ± 2.45	30.0 ± 1.46	0.20 ± 2.04	1.07 ± 2.34		
Sig. bet. grps.	p_1_ < 0.001^*^, p_2_ < 0.001^*^, p_3_ < 0.001^*^, p_4_ < 0.001^*^, p_5_ < 0.001^*^, p_6_ = 0.676					
AD						
Min. – Max.	17.0–26.0	56.0–63.0	-3.0–5.0	-4.0–4.0	2136.403	< 0.001^*^
Mean ± SD.	21.07 ± 2.71	60.53 ± 1.88	1.13 ± 2.36	0.93 ± 2.37		
Sig. bet. grps.	p_1_ < 0.001^*^, p_2_ < 0.001^*^, p_3_ < 0.001^*^, p_4_ < 0.001^*^, p_5_ < 0.001^*^, p_6_ = 0.995					
AC						
Min. – Max.	21.0–30.0	29.0–31.0	-2.0–5.0	-1.0–3.0	1001.555	< 0.001^*^
Mean ± SD.	25.27 ± 2.74	30.33 ± 0.72	1.20 ± 2.34	0.33 ± 1.18		
Sig. bet. grps.	p_1_ < 0.001^*^, p_2_ < 0.001^*^, p_3_ < 0.001^*^, p_4_ < 0.001^*^, p_5_ < 0.001^*^, p_6_ = 0.610					
BD						
Min. – Max.	18.0–27.0	29.0–33.0	-2.0–5.0	-3.0–4.0	762.459	< 0.001^*^
Mean ± SD.	22.73 ± 2.66	30.87 ± 1.19	1.27 ± 2.52	0.80 ± 1.86		
Sig. bet. grps.	p_1_ < 0.001^*^, p_2_ < 0.001^*^, p_3_ < 0.001^*^, p_4_ < 0.001^*^, p_5_ < 0.001^*^, p_6_ = 0.932					

F: F for One-way ANOVA test, pairwise comparison bet. each 2 groups were done using Post Hoc Test (Tukey); p: p value for comparing between the studied groups; p_1_: p value for comparing between Group I and Group II; p_2_: p value for comparing between Group I and Group III; p_3_: p value for comparing between Group I and Group IV; p_4_: p value for comparing between Group II and Group III; p_5_: p value for comparing between Group II and Group IV; p_6_: p value for comparing between Group III and Group IV; *: Statistically significant at *p* ≤ 0.05; Group I: C2mm; Group II: C4mm; Group III: D2mm. Group IV: D4mm

The article "Effect of soft tissue thickness on accuracy of conventional and digital implant impression techniques" was published in 2024. Journal: BMC Oral Health.

### Effect of soft tissue thickness on accuracy of impression for implant restorations

A. Using the conventional impression technique, Table 3 illustrates that there was a significant difference between groups I and II (C2mm and C4mm) of six distances between implant analogues, with a p value of p1 < 0.001. In group I (C2mm), the mean difference between six distances after subtracting from their reference model (I) was AB (28.93 ± 2.99), BC (-8.07 ± 3.01), CD (19.53 ± 2.45), AD (21.07 ± 2.71), AC (25.27 ± 2.74), BD (22.73 ± 2.66). This is less than the mean difference of six distances in group II (C4mm) after subtracting from their reference model (2), AB (49.47 ± 1.06), BC (39.47 ± 1.36), CD (30.0 ± 1.46), AD (60.53 ± 1.88), AC (30.33 ± 0.72), BD (30.87 ± 1.19). This indicates that increasing soft tissue thickness reduces the accuracy of conventional implant impression.
B. In digital impression technique: comparison between groups III, IV (D2mm, D4mm):

In comparison between group III (D2mm) and group IV (D4mm) of six distances between implant analogues there was no significant difference between them, p value was more than 0.001 where AB (p_6_ = 0.410), BC (p_6_ = 0.580), CD (p_6_ = 0.676), AD (p_6_ = 0.676), AC (p_6_ = 0.610) and BD (p_6_ = 0.932). which means that the thickness of soft tissue has no effect on accuracy of digital impression for implant restoration.

### Conventional impression versus digital impression

#### Comparison between groups I, III (C2mm, D2mm)

p value was p1 < 0.001, as indicated in Table (2), indicating a significant difference between group I (C2mm) and group III (D2mm) of six distances between implant analogs. This suggests that the impression technique affects accuracy. Ingroup I (C2mm), the mean difference between six distances after subtracting from their reference model (1) was AB (28.93 ± 2.99), BC (-8.07 ± 3.01), CD (19.53 ± 2.45), AD (21.07 ± 2.71), AC (25.27 ± 2.74), BD (22.73 ± 2.66). This was greater than the mean difference of group III (D2mm), which was AB (-0.93 ± 2.12), BC (-1.53 ± 2.97), CD (0.20 ± 2.04), AD (1.13 ± 2.36), AC (1.20 ± 2.34), BD (1.27 ± 2.52).

The article "Effect of soft tissue thickness on accuracy of conventional and digital implant impression techniques" was published in 2024. Journal: BMC Oral Health.

#### Comparison between groups II, IV (C4mm, D4mm)

There was a significant difference between group II (C4mm) and group IV (D4mm) of six distances between implant analogues; the p-value was p1 < 0.001, indicating that the accuracy of the impression is influenced by the impression technique. Group II (C4mm) had mean differences after subtracting from their reference model (2) of AB(49.47 ± 1.06), BC (39.47 ± 1.36), CD (30.0 ± 1.46), AD(60.53 ± 1.88), AC(30.33 ± 0.72), and BD(30.87 ± 1.19). These were greater than mean differences of group IV (D4mm) after subtracting from their reference model (2) of AB(0.33 ± 2.29), BC (-0.47 ± 1.06), CD (1.07 ± 2.34), AD(0.93 ± 2.37), AC(0.33 ± 1.18), BD(0.80 ± 1.86). This shows that digital impression techniques are more accurate than conventional techniques.

## Discussion

An impression that accurately record the three-dimensional implant placements is necessary in order to produce a prosthesis that fits passively [1].

Because epoxy resin models are more stable than plaster models and have an elastic modulus that is acceptable for a material that is analogous to bone [9–11], they were utilized as reference models in this work.

In order to replicate the soft tissues and residual ridge mucosa in epoxy resin models, flexible polyurethane material with a hardness of 65 N/mm2 was applied. This allowed for equivalent results when the implant depth factor was assessed, as it was done by Taduri et al., [11]

Internal connection system were placed because of their benefits, which include easier abutment connection, increased stability, anti-rotation, greater resistance to lateral loads, and improved force distribution [14].

The original implants and their laboratory analogues had a significantly different scanbody fit, according to Stimmelmayr et al. [15], whose findings were taken into account in our study.

In each model, which has a varied mucosal thickness (2 mm, 4 mm), the four implant analogues were positioned parallel to each other to mimic typical clinical scenarios where implants may need to be implanted in canine and lower molar areas. This was in line with certain research [16], which suggested that less impression coping above the gingival margin and more below it could reduce the stability of impression coping in the impression material and affect impression accuracy for conventional impression [13].

In addition to the depth in digital impressions that was previously mentioned, Giménez-González et al. placed the implant equigingivally (2 and 4 mm subgingivally) and stated that the depth of the implant should be taken into consideration when choosing the ISB design because the amount of visible scanbody influences the accuracy of digital impressions [17].

The article "Effect of soft tissue thickness on accuracy of conventional and digital implant impression techniques" was published in 2024. Journal: BMC Oral Health.

Impressions were taken at the implant level in this in-vitro study because it makes it easier to choose and adjust abutments and prostheses. This is in agreement with Choi et al., [18], Daoudi et al., [19] and Lee et al., [20].

Many authors examined and compared the accuracy of direct and indirect methods; a few of them came to the conclusion that the direct method was more accurate. In this study, the direct unsplinted impression technique was used [22–24]. A previous study found that the direct technique was more accurate when there were more than three implants, but there was no discernible difference between the direct and indirect techniques when there were three or fewer implants. A few others discovered that the non-splinting method was more precise than the splinting methods [26–29]. These disparate outcomes could be attributed to variations in the materials, operators, and methodology.

In the current study, adhesive material was used in accordance with the suggestions made by Vigolo et al. (2000), (2003), and (2004) that it was important to prevent coping movement, particularly when screwing or unscrewing the coping screw and to provide intimate contact between coping and impression material [31–33]. Polyvinylsiloxane (PVS) was chosen as the impression material for this study because it exhibits accuracy and enough rigidity when holding the imprint coping to avoid undesired displacement [33]. They have the least amount of distortion of any impression material, good elastic recovery from undercuts, and sufficient tear strength. (34–37). Dental stone certified by the ADA as type IV was used to pour all impressions.

According to Arcuri et al. [40], In this study’s digital scanning, PEEK ISB (cylindrical design with beveled upper section) was used because The most accurate material was PEEK; titanium and hybrid PEEK with titanium came next. Since the fit of these scanbodies on implants determines accuracy, an extra oral laboratory scanner was used in this study. Laboratory scanning on the stone cast would result in fewer inaccuracies because Stimmelmayer et al. reported an average disparity in the fit of scanbodies of 39 μm on the original implants and only 11 μm on implant analogues [15, 41].

For this in-vitro study, laboratory scanners were required since scanning multiple implants in an edentulous jaw could create specific difficulties. The intraoral scanner may find it difficult to distinguish between the several similar scan bodies being used and, consequently, to locate the correct location in the jaw [42]. which is corroborated by several investigations [40, 43–45]. Su and Ting-Shu also noted that the IOS precision was significantly lower and divergence increased with the number of scanned teeth when laboratory data were compared [46]. Because all scanbodies are identical and there are no anatomical landmarks, completing an edentulous jaw scan could be challenging. Multiple difficulties are found when two implants are scanned, according to numerous research [47].

The article "Effect of soft tissue thickness on accuracy of conventional and digital implant impression techniques" was published in 2024. Journal: BMC Oral Health.

Extra oral scanner with all-in-one process (stable scan stage method) were used in this study in which camera moved around the model which is stable during scanning unlike conventional scanner in which we need to mount model with fixture or clays they are not tedious but also time consuming.

This in-vitro study uses a one-step strategy or technique to scan the model and ISBs all at once in order to increase accuracy which was similar to what reported in study of Motel et al., when the model is scanned twice, once without ISBs and once with ISBs placed on the model, in comparison to one step and two step scanning methods [48].

Measuring microscopes, strain gauges, Vernier calipers, micrometers, and other instruments could only measure in two dimensions when used in impression techniques [49].However, significant data is lost when measurements are limited to two dimensions. The CMM, or coordinate measuring machine, was thus utilized in this study’s measurement process since it enables the evaluation of distortion in three dimensions. A 3D magnitude represents the distance between two points when the displacement between them is measured along all three axes (X, Y, and Z). It is possible to record the rotational displacement of the hex and the 3D orientation of analogs when points from various implant casts have a common reference inside a coordinate system [49]. This was consistent with some recent research [29, 39, 50].

The result of this in-vitro study showed that there was significant difference in accuracy between different soft tissue thickness in conventional impression techniques (direct unsplinted technique). these results agreed with several studies showing that the deeper an implant is placed subgingivally, the less area of the impression coping will be covered by impression material and the impression will be less accurate [7].

Additionally, in line with a study that employed silicone gingival masks on all of the master models, which accurately modeled the soft tissues A comparison of the linear and angular aspects of master models with laboratory analogues positioned deeper within the gingival mask revealed statistically significant differences [11]. The Linkevicius et al. study also mentioned that the subgingival position of implants had an impact on impression accuracy. This could have to do with how long the impression coping is embedded in the impression [51, 52]. Additionally, it has been discovered that placing dental implants deeply reduces the stability of the impression coping, which has an immediate impact on recording implant position. Concerning the depth of the implant and tissue thickness. These results are in agreement with several studies showing that implant depth and tissue thickness had no significant effect in digital scanning [16, 47, 54, 55].

The article "Effect of soft tissue thickness on accuracy of conventional and digital implant impression techniques" was published in 2024. Journal: BMC Oral Health.

Additionally, in agreement with Arcuri et al., concluded that implant depth had no effect on the ultimate accuracy of digital impressions when the influence of implant depth using digital impression had been studied by placing the implants equigingivally (3 and 6 mm).

subgingivally [40]. so the first null hypothesis is there were no significant differences in accuracy of implant level impressions of different tissue thickness and subgingval depths of implant is accepted in digital impression.

This in-vitro study, however, varies from prior research in that it is directly related to scanbody visibility, which may impair accuracy, whereas other research takes implant depth into consideration. When the scanbody is fully visible, determining the implant position becomes less error-prone; hence, the deeper the implant, the longer the scanbody should be placed [17, 56, 57]. Furthermore, this study differs from another by Giménez-González et al. that examined implants positioned equigingivally (2 and 4 mm subgingivally) and suggested that the implant depth should be taken into account when selecting the ISB design because the amount of visible ISB affects the accuracy of digital impressions [17].

As a result, the second null hypothesis that the digital impression would provide accuracy comparable to the conventional technique in complete arch cases was rejected based on the specific results of this in-vitro study conducted with a specific scanner under a specific set of conditions and without a significant difference in implant position accuracy.

These results are in line with multiple studies that proved that digital impressions were more accurate than conventional impressions [58–63].

However, the results are in disagreement with studies showing that no difference in accuracy between digital and conventional method [56].

On the other hand, this in-vitro study not parallel with other research which concluded that conventional impression is more accurate than digital impression [64–67].

The article "Effect of soft tissue thickness on accuracy of conventional and digital implant impression techniques" was published in 2024. Journal: BMC Oral Health.

The limitations of this in-vitro study are that the procedure has not been done under clinical condition, used only one type of implant connection and were tested using single impression material and single digital impression technique.

## Conclusions

Within the limitations of this in-vitro study the digital impressions provided more accurate outcome with implant placed deeper in soft tissue than conventional impressions. Also, it appears that the digital impression techniques reproduced the three-dimensional position of implants more accurately than conventional techniques.

## Data Availability

The datasets used and/or analyzed during the current study are available from the corresponding author upon reasonable request.

## Declarations

### Clinical trial number

it is an in-vitro study.

## Abbreviations

3-D: 3-Dimensional
PVS: Polyvinylsiloxanes
IOSs: Intraoral Scanners
ISB: Intra-Oral Scan Body
CAD: Computer-Aided Design
PEEK: Polyetheretherketone
DIIs: Digital Implant Impressions
LF: Library Files
ME: Mesh
AGD: Auxiliary Geometric Device
CAD/CAM: Computer-Aided Design and Manufacturing
CMM: Co-ordinate Measuring Machines
STL: Surface Tessellation Language
CAE: Computer-Aided Engineering
REC: Research Ethics Committee

## References

[1] Arikan H, Muhtarogullari M, Uzel SM, Guncu MB, Aktas G, Marshall LS, Turkyilmaz I. Accuracy of digital impressions for implant-supported complete-arch prosthesis when using an auxiliary geometry device. J Dent Sci. 2023;808–13.10.1016/j.jds.2023.01.012PMC1006848937021239

[2] Pjetursson BE, Thoma D, Jung R, Zwahlen M, Zembic A. A systematic review of the survival and complication rates of implant-supported fixed dental prostheses (FDP s) after a mean observation period of at least 5 years. Clin Oral Implants Res. 2012;23:22–38.23062125 10.1111/j.1600-0501.2012.02546.x

[3] Buzayan MM, Yunus NB. Passive Fit in Screw retained multi-unit Implant Prosthesis understanding and achieving: a review of the literature. J Indian Prosthodont Soc. 2014;16–23.10.1007/s13191-013-0343-xPMC393503724604993

[4] Abduo J, Bennani V, Waddell N, Lyons K, Swain M. Assessing the fit of implant fixed prostheses: a critical review. Int J Oral Maxillofac Implants. 2010;25(3):506–15.20556249

[5] Eliasson A, Örtorp A. The accuracy of an implant impression technique using digitally coded healing abutments. Clin Implant Dent Relat Res. 2012;14:e30–8.21453396 10.1111/j.1708-8208.2011.00344.x

[6] Hale A, Mehmet M, Sema M, Mustafa B, Lindsay S. Accuracy of digital impressions. For implant-supported complete-arch prosthesis when using an auxiliary geometry device. J Dent Sci.2023(18): 808–13.10.1016/j.jds.2023.01.012PMC1006848937021239

The article "Effect of soft tissue thickness on accuracy of conventional and digital implant impression techniques" was published in 2024. Journal: BMC Oral Health.

[7] Lee H, Ercoli C, Funkenbusch PD, Feng C. Effect of subgingival depth of implant placement on the dimensional accuracy of the implant impression: an in vitro study. J Prosthet Dent. 2008;99(2):107–13.18262011 10.1016/S0022-3913(08)60026-8

[8] Richi MW, Kurtulmus-Yilmaz S, Ozan O. Comparison of the accuracy of different impression procedures in case of multiple and angulated implants. Head Face Med. 2020;(16) 9.10.1186/s13005-020-00225-3PMC719714832366261

[9] Al Quran FA, Rashdan BA, Abu Zomar AA, Weiner S. Passive fit and accuracy of three dental implant impression techniques. Quintessence Int. 2012;43(2):119–25.22257873

[10] Lee CK, Karl M, Kelly JR. Evaluation of test protocol variables for dental implant fatigue research. Dent Mater. 2009;25(11):1419–25.19646746 10.1016/j.dental.2009.07.003

[11] Taduri T, Mathur S, Upadhyay S, Patel K, Shah M. Effect of Implant Angulation and depth on the Accuracy of casts using the Open Tray Splinted impression technique. Oral Implantol. 2021;47(6):447–54.10.1563/aaid-joi-D-19-0024633270885

[12] Sorrentino R, Gherlone EF, Calesini G, Zarone F. Effect of implant angulation, connection length, and impression material on the dimensional accuracy of implant impressions: an in vitro comparative study. Clin Implant Dent Relat Res. 2010;12:e63–76.19438937 10.1111/j.1708-8208.2009.00167.x

[13] Hazboun GBA, Masri R, Romberg E, Kempler J, Driscoll CF. Effect of implant angulation and impression technique on impressions of NobelActive implants. J Prosthet Dent. 2015;113(5):425–31.25749089 10.1016/j.prosdent.2014.10.009

[14] Gehrke P, Rashidpour M, Sader R, et al. A systematic review of factors impacting intraoral scanning accuracy in implant dentistry with emphasis on scan bodies. Int J Implant Dent. 2024;10:20.38691258 10.1186/s40729-024-00543-0PMC11063012

[15] Stimmelmayr M, Güth J-F, Erdelt K, Edelhoff D, Beuer F. Digital evaluation of the reproducibility of implant scanbody fit—an in vitro study. Clin Oral Investig. 2012;16(3):851–6.21647591 10.1007/s00784-011-0564-5

[16] Giménez B, Özcan M, Martínez-Rus F, Pradíes G. Accuracy of a digital impression system based on active triangulation technology with blue light for implants: effect of clinically relevant parameters. Implant Dent. 2015;24(5):498–504.26057777 10.1097/ID.0000000000000283

[17] Gimenez-Gonzalez B, Hassan B, Özcan M, Pradíes G. An in vitro study of factors influencing the performance of digital intraoral impressions operating on active wavefront sampling technology with multiple implants in the edentulous maxilla. J Prosthodont. 2017;26(8):650–5.26934046 10.1111/jopr.12457

The article "Effect of soft tissue thickness on accuracy of conventional and digital implant impression techniques" was published in 2024. Journal: BMC Oral Health.

[18] Choi J-H, Lim Y-J, Kim C-W. Evaluation of the accuracy of implant-level impression techniques for internal-connection implant prostheses in parallel and divergent models. Int J Oral Maxillofac Implants. 2007;22(5):761–8.17974110

[19] Daoudi MF, Setchell DJ, Searson LJ. An evaluation of three implant level impression techniques for single tooth implant. Eur J Prosthodont Restor Dent. 2004;12(1):9–14.15058176

[20] Lee Y-J, Heo S-J, Koak J-Y, Kim S-K. Accuracy of different impression techniques for internal-connection implants. Int J Oral Maxillofac Implants. 2009;24(5):823–30.19865622

[21] Bartlett DW, Greenwood R, Howe L. The suitability of head-of-implant and conventional abutment impression techniques for implant-retained three unit bridges: an in vitro study. Eur J Prosthodont Restor Dent. 2002;10(4):163–6.12526273

[22] Assuncao WG, Gennari Filho H, Zaniquelli O. Evaluation of transfer impressions for osseointegrated implants at various angulations. Implant Dent. 2004;13(4):358–66.15591998 10.1097/01.id.0000144509.58901.f7

[23] Akca K, Çehreli MC. Accuracy of 2 impression techniques for ITI implants. Int J Oral Maxillofac Implants. 2004;19(4):517–23.15346748

[24] Lee H, So JS, Hochstedler J, Ercoli C. The accuracy of implant impressions: a systematic review. J Prosthet Dent. 2008;100(4):285–91.18922257 10.1016/S0022-3913(08)60208-5

[25] Ahumada-DeGirolamo D, Azocar A, Delpiano-Mesina C, Maldonado-Cortés P, Muñoz MA, Luque-Martínez I, Bravo-Gallardo F. Splinting or non-splinting of fixed prostheses on adjacent implants: a critical review. J Prosth Res. 2023;2:206–14.10.2186/jpr.JPR_D_22_0022037648482

[26] AL-Juboori MJ, AL-Attas MA, Minichetti J, Akhikar J. (2024). The Use of Splinted Versus Nonsplinted Prosthetic Design in Dental Implants: A Literature Review. J.Oral Implantology.2024; (1): 50–64.10.1563/aaid-joi-D-23-0007738329841

[27] Burawi G, Houston F, Byrne D, Claffey N. A comparison of the dimensional accuracy of the splinted and unsplinted impression techniques for the bone-lock implant system. J Prosthet Dent. 1997;77(1):68–75.9029468 10.1016/s0022-3913(97)70209-9

[28] Mostafa TMN, Elgendy MNM, Kashef NA, Halim MM. Evaluation of the precision of three implant transfer impression techniques using two elastomeric impression materials. Int J Prosthodont. 2010;23(6):525–8.21209987

[29] Vojdani M, Torabi K, Ansarifard E. Accuracy of different impression materials in parallel and nonparallel implants. J Dent Res. 2015;12(4):315.10.4103/1735-3327.161429PMC453318826288620

[30] Vigolo P, Fonzi F, Majzoub Z, Cordioli G. An evaluation of impression techniques for multiple internal connection implant prostheses. J Prosthet Dent. 2004;92(5):470–6.15523336 10.1016/j.prosdent.2004.08.015

The article "Effect of soft tissue thickness on accuracy of conventional and digital implant impression techniques" was published in 2024. Journal: BMC Oral Health.

[31] Vigolo P, Majzoub Z, Cordioli G. In vitro comparison of master cast accuracy for single-tooth implant replacement. J Prosthet Dent. 2000;83(5):562–6.10793389 10.1016/s0022-3913(00)70015-1

[32] Vigolo P, Majzoub Z, Cordioli G. Evaluation of the accuracy of three techniques used for multiple implant abutment impressions. J Prosthet Dent. 2003;89(2):186–92.12616240 10.1067/mpr.2003.15

[33] Moreira AH, Rodrigues NF, Pinho AC, Fonseca JC, Vilaça JL. Accuracy comparison of implant impression techniques: a systematic review. Clin Implant Dent Relat Res. 2015;17:e751–64.25828851 10.1111/cid.12310

[34] Tabesh M, Alikhasi M, Siadat H. A comparison of implant impression precision: different materials and techniques. J Clin Experimental Dentistry. 2018;2018(2):e151.10.4317/jced.54457PMC589979829670733

[35] Wassell R, Barker D, Walls A. Crowns and other extra-coronal restorations: impression materials and technique. Br Dent J. 2002;192(12):679–90.12125794 10.1038/sj.bdj.4801456

[36] Nissan J, Laufer B-Z, Brosh T, Assif D, Maurice T. Accuracy of three polyvinyl siloxane putty-wash impression techniques. J Prosthet Dent 2000;83(2):161-5.10.1016/s0022-3913(00)80007-410668027

[37] Palantza E, Sykaras N, Zoidis P. Kourtis S. In vitro comparison of accuracy between conventional and digital impression using elastomeric materials and two intra-oral scanning devices. J Esthet Restor Dent. 2024;1-20.10.1111/jerd.1322738534043

[38] Martínez-Rus F, García C, Santamaría A, Özcan M, Pradíes G. Accuracy of definitive casts using 4 implant-level impression techniques in a scenario of multi-implant system with different implant angulations and subgingival alignment levels. Implant Dent. 2013;22(3):268–76.23615660 10.1097/ID.0b013e3182920dc5

[39] Geramipanah F, Sahebi M, Davari M, Hajimahmoudi M, Rakhshan V. Effects of impression levels and trays on the accuracy of impressions taken from angulated implants. Clin Oral Implants Res. 2015;26(9):1098–105.24934081 10.1111/clr.12410

[40] Arcuri L, Pozzi A, Lio F, Rompen E, Zechner W, Nardi A. Influence of implant scanbody material, position and operator on the accuracy of digital impression for complete-arch: a randomized in vitro trial. J Prosthodont Res. 2020;64(2):128–36.31255546 10.1016/j.jpor.2019.06.001

[41] Andriessen FS, Rijkens DR, Van Der Meer WJ, Wismeijer DW. Applicability and accuracy of an intraoral scanner for scanning multiple implants in edentulous mandibles: a pilot study. J Prosthet Dent. 2014;111(3):186–94.24210732 10.1016/j.prosdent.2013.07.010

[42] Flügge TV, Att W, Metzger MC, Nelson K. Precision of Dental Implant Digitization using Intraoral scanners. Int J Prosthodont. 2016;29(3):277–83.27148990 10.11607/ijp.4417

The article "Effect of soft tissue thickness on accuracy of conventional and digital implant impression techniques" was published in 2024. Journal: BMC Oral Health.

[43] Keul C, Güth J-F. Accuracy of full-arch digital impressions: an in vitro and in vivo comparison. Clin Oral Investig. 2020;24(2):735–45.31134345 10.1007/s00784-019-02965-2

[44] Mangano F, Gandolfi A, Luongo G, Logozzo S. Intraoral scanners in dentistry: a review of the current literature. BMC Oral Health. 2017;17(1):1–11.10.1186/s12903-017-0442-xPMC572769729233132

[45] Patzelt SB, Vonau S, Stampf S, Att W. Assessing the feasibility and accuracy of digitizing edentulous jaws. J Am Dent Assoc. 2013;144(8):914–20.23904578 10.14219/jada.archive.2013.0209

[46] Su T-s, Sun J. Comparison of repeatability between intraoral digital scanner and extraoral digital scanner: an in-vitro study. J Prosthodont Res. 2015;59(4):236–42.26211702 10.1016/j.jpor.2015.06.002

[47] Giménez B, Özcan M, Martínez-Rus F, Pradíes G. Accuracy of a digital impression system based on parallel confocal laser technology for implants with consideration of operator experience and implant angulation and depth. Int J Oral Maxillofac Implants. 2014;29(4):853–62.25032765 10.11607/jomi.3343

[48] Motel C, Kirchner E, Adler W, Wichmann M, Matta RE. Impact of different scan bodies and scan strategies on the accuracy of digital implant impressions assessed with an intraoral scanner: an in vitro study. J Prosthodont. 2020;29(4):309–14.31802574 10.1111/jopr.13131

[49] Hoist S, Blatz MB, Bergler M, Goellner M, Wichmann M. Influence of impression material and time on the 3-dimensional accuracy of implant impressions. Quintessence Int. 2007;38(1):67–73.17216911

[50] Tsagkalidis G, Tortopidis D, Mpikos P, Kaisarlis G, Koidis P. Accuracy of 3 different impression techniques for internal connection angulated implants. J Prosthet Dent. 2015;114(4):517–23.26213265 10.1016/j.prosdent.2015.05.005

[51] Linkevicius T, Svediene O, Vindasiute E, Puisys A, Linkeviciene L. The influence of implant placement depth and impression material on the stability of an open tray impression coping. J Prosthet Dent. 2012;108(4):238–43.23031730 10.1016/S0022-3913(12)60169-3

[52] Öngül D, Gökçen-Röhlig B, Şermet B, Keskin, HJAdj. A comparative analysis of the accuracy of different direct impression techniques for multiple implants. Aust Dent J. 2012;57(2):184–9.22624759 10.1111/j.1834-7819.2012.01685.x

[53] Beyabanaki E, Shamshiri AR, Alikhasi M, Monzavi AJJP. Effect of splinting on dimensional accuracy of impressions made of implants with different subgingival alignments. J Prosthodont. 2017;26(1):48–55.26436559 10.1111/jopr.12368

[54] Giménez B, Özcan M, Martínez-Rus F, Pradíes G. Accuracy of a digital impression system based on active wavefront sampling technology for implants considering operator experience, implant angulation, and depth. Clin Implant Dent Relat Res. 2015;17:e54–64.23879869 10.1111/cid.12124

The article "Effect of soft tissue thickness on accuracy of conventional and digital implant impression techniques" was published in 2024. Journal: BMC Oral Health.

[55] Giménez B, Pradíes G, Martínez-Rus F, Özcan M. Accuracy of two digital implant impression systems based on confocal microscopy with variations in customized software and clinical parameters. Int J Oral Maxillofac Implants. 2015;30(1):56–64.25615916 10.11607/jomi.3689

[56] Papaspyridakos P, Gallucci GO, Chen CJ, Hanssen S, Naert I, Vandenberghe B. Digital versus conventional implant impressions for edentulous patients: accuracy outcomes. Clin Oral Implants Res. 2016;27(4):465–72.25682892 10.1111/clr.12567

[57] Gherlone E, Capparé P, Vinci R, Ferrini F, Gastaldi G, Crespi R. Conventional Versus Digital impressions for all-on-four restorations. Int J Oral Maxillofac Implants. 2016;31(2):324–30.27004280 10.11607/jomi.3900

[58] Alikhasi M, Siadat H, Nasirpour A, Hasanzade M. Three-dimensional accuracy of digital impression versus conventional method: effect of implant angulation and connection type. Int J Dent. 2018;2018:3761750.29971107 10.1155/2018/3761750PMC6008832

[59] Albayrak B, Sukotjo C, Wee AG, Korkmaz İH, Bayındır F. Three-Dimensional Accuracy of Conventional Versus Digital Complete Arch Implant impressions. J Prosthodont. 2021;30(2):163–70.32935894 10.1111/jopr.13264

[60] Menini M, Setti P, Pera F, Pera P, Pesce P. Accuracy of multi-unit implant impression: traditional techniques versus a digital procedure. Clin Oral Investig. 2018;22(3):1253–62.28965251 10.1007/s00784-017-2217-9

[61] Amin S, Weber HP, Finkelman M, El Rafie K, Kudara Y, Papaspyridakos P. Digital vs. conventional full-arch implant impressions: a comparative study. Clin Oral Implants Res. 2017;28(11):1360–7.28039903 10.1111/clr.12994

[62] Farhan F-A, Ali-Jameel-Abdul Sahib A-A. Comparison of the accuracy of intraoral digital impression system and conventional impression techniques for multiple implants in the full-arch edentulous mandible. J Clin Experimental Dentistry. 2021;13(5):e487.10.4317/jced.57926PMC810693933981396

[63] Papaspyridakos P, Vazouras K, Chen Yw, Kotina E, Natto Z, Kang K, et al. Digital vs conventional implant impressions: a systematic review and meta-analysis. J Prosthodont. 2020;29(8):660–78.32613641 10.1111/jopr.13211

[64] Alsharbaty MHM, Alikhasi M, Zarrati S, Shamshiri AR. A clinical comparative study of 3-dimensional accuracy between digital and conventional implant impression techniques. J Prosthodont. 2019;28(4):e902–8.29423969 10.1111/jopr.12764

[65] Huang R, Liu Y, Huang B, Zhang C, Chen Z, Li Z. Improved scanning accuracy with newly designed scan bodies: an in vitro study comparing digital versus conventional impression techniques for complete-arch implant rehabilitation. Clin Oral Implants Res. 2020;31(7):625–33.32181919 10.1111/clr.13598

The article "Effect of soft tissue thickness on accuracy of conventional and digital implant impression techniques" was published in 2024. Journal: BMC Oral Health.

[66] Pachiou A, Zervou E, Tsirogiannis P, Sykaras N, Tortopidis D, Kourtis S. Characteristics of intraoral scan bodies and their influence on impression accuracy: a systematic review. J Esthet Restor Dent. 2023;1–13.10.1111/jerd.1307437381677

[67] Ahn G-Z, Lee J-S. Comparison of the accuracy of implant digital impression coping. J Dent Rehabil Appl Sci. 2020;36:29–40.

